This article has been retracted.

# Data analysis and personalized recommendation of western music history information using deep learning under Internet of Things

**DOI:** 10.1371/journal.pone.0262697

**Published:** 2022-01-26

**Authors:** Zongye Yang

**Affiliations:** School of Music, Drama and Dance, The Herzen State Pedagogical University of Russia, St.Petersburg, Russia; Ministry of Natural Resources North Sea Bureau, CHINA

## Abstract

To improve the teaching effect of western music history, the curriculum reform of history education needs to be promoted under the background of the Internet of Things (IoT). At first, a discussion is made on the characteristics of history course, which is combined with the characteristics of teaching data easy to collect under the background of IoT. An analysis is conducted on the related theory of educational data mining. Then, the concept of personalized recommendation is proposed based on deep learning (DL) algorithm. Finally, online and offline experiments are designed to verify the performance of the algorithm from review and investigation, smoothness, and participation of difficulty. The research results show that in terms of offline recommendation accuracy, the average record length in Math data set is 24.5, which is much smaller than that in range data set. The research has obvious innovation significance compared with other studies. In the process of target review and investigation, it is found that the research method here involves a wider range of knowledge and higher reliability. In terms of the difficulty of recommending questions, the Deep Reinforcement Exercise (DRE) recommendation algorithm can adaptively adjust the difficulty of recommending questions. It also allows students to set different learning goals through participation goals. But in the experiments on Math data set, Step 10’s recommendation results are not very good, and the difficulty level varies greatly. If the goal setting is high, the problem recommended to students is too difficult, students may answer these questions wrongly, forcing the algorithm to adjust the difficulty adaptively. According to the above results, DRE recommendation algorithm can adapt to different learning needs and customize the recommendation results, thus opening up a new path for the teaching of western music history. Besides, the combination of DL algorithm and western music history teaching design can recommend learning materials, which is of great significance in the teaching of history courses.

## Introduction

With the rapid development of computer communication technology, changes in all walks of life are developing with each passing day. Convenient communication conditions have brought massive knowledge bases, thus laying a solid foundation for the reform of network teaching [1]. The change of teaching concept is essentially the change of teaching thinking driven by the development of network technology. The development of communication technology makes all fields of information common, and promotes the integration and exchange of eastern and western cultural information [2]. In this context, constructing a new paradigm of western music history teaching thinking is conducive to the combination of learning and thinking, sensing and reflection, to develop the creativity of teachers and students and produce new ways of thinking and conscious pursuit [3]. Although there is no new teaching method in western history education, many studies have provided technical support for it.

Huang (2021) pointed out that in recent years, with the deepening of teaching reform and the wide application of modern information technology, how to combine the traditional teaching of western music history and masterpiece appreciation course with network multimedia means had become a topic worthy of further discussion [4]. Lee (2020) thought that network teaching should be based on traditional teaching and assisted by multimedia teaching. In terms of function, it is more to make up for the shortcomings of traditional teaching and multimedia courseware-assisted teaching, and play a certain role in teaching supervision. Relying on the network platform, the excellent classroom videos and multimedia courseware can be updated in time to realize the sharing of network information resources [5]. Edwards and Cheok (2018) reckoned that the construction and application of network video teaching platform had made the level of teaching reform in China more in-depth. Combined with the use of modern information technology, the level of education has been improved intelligently. How to organically combine the course of western music history and masterpiece appreciation with modern scientific and technological means requires extensive practitioners to actively practice and conduct in-depth discussions, thus improving the teaching level qualitatively [6]. Daniel (2019) noticed that the network was frequently used in the teaching of various courses, which brought vitality to the teaching of western music history. Compared with traditional teaching, what new teaching methods can be applied to teaching after the network intervention and where the advantages of network teaching compared with traditional teaching are the focus of the current research on western music history teaching [7]. Shin (2021) reckoned that in the context of the rapid development of the Internet in the 21st century and the comprehensive extension of the network to all corners of modern life, the original teaching ideas, methods and means must change accordingly. Otherwise, they will not be able to connect with the new situations and new problems in the teaching field under the existing conditions. Hence, teachers should be able to carry out targeted teaching [8]. Torshizi and Bahraman (2019) signified that deep learning was a research field that had attracted much attention in recent years and played an important role in machine learning (ML). If the shallow learning is a wave of ML, DL, as a new field of ML, will set off another wave. DL realizes the feature extraction of external input data from low level to high level by establishing and simulating the hierarchical structure of human brain, to explain external data [9].

In summary, the present work initially explores the data of modern education, optimizes the western music history, and explores and proposes a personalized recommendation teaching system. Then, the personalized recommendation system is upgraded based on DL. Different from other studies, the present work has changed the existing teaching mode of western music history and comprehensively upgraded it through the optimized personalized recommendation system. The teaching of western music history is reformed according to the traditional network teaching, which is combined with the network teaching and DL algorithm to optimize the personalized recommendation system. A new way is opened up for the teaching of western music history, and contributions are made to the reform of traditional teaching mode.

## Educational theories and personalized recommendation system

### Research of educational data mining

With the fast growth of information technology, education and learning can break through the limitations of time and space. With the significant expansion of data collection methods, the data accumulation in education practices has also increased. Educational data mining (EDM) is becoming an increasingly independent research direction, which has attracted the attention of researchers in psychology, computer, statistics, pedagogy and other fields [10, 11]. White (2019) found that data-accorded portraying of learner models, generation of effective learning support, learning behavior patterns and characteristics, learning performance prediction, learning feedback, and evaluation have become the research hotspots of teaching methods [12]. Generally, the definition of EDM is that using data mining technology and data analysis methods to analyze different types of educational data to provide educational research and services. The sources of data for analysis and mining are online and offline. Fig 1 displays the primary contents and fields of EDM research.

**Fig 1:** Primary research fields of EDM.

As shown in Fig 1, EDM includes six basic research areas, i.e., the visualization of educational data, management and evaluation of learning resources, personalized recommendation of learning resources, analysis of students’ social ability, construction of educational knowledge map, and analysis of modeling and cognitive ability of students. The goal of educational data visualization is to screen useful information and important data results in the data for education optimization, and take the data as a reference for relevant decision-making [13, 14]. Statistical analysis and data analysis are common methods of educational data visualization. Learning resources represent the infrastructure related to teaching and learning processes, such as textbooks, tutorials, exercises, course videos, and knowledge systems [15, 16]. On the one hand, the effective evaluation of learning resources can help teachers and students understand the quality of learning content. On the other hand, it can assist online system administrators in managing different types of resources and providing efficient search services. The purpose of individual modeling of students is to explain the characteristics of students through different levels of information, including the daily performance, learning habits, internal knowledge, learning ability, learning interest, and mental health level of students [17, 18]. Student modeling is the emphasis of EDM, because the modelling results can support various educational applications, such as performance prediction, and resource recommendation. Personalized recommendation is a momentous way to realize personalized learning, aimed at offering personalized learning recommendation services such as learning activities, behavior activity records, consumption records, course recommendations, and sports recommendations. Diversified data mining technologies can be applied to personalized recommendation, including classification and regression, model mining, sequence analysis, and recommendation algorithms [19]. The analysis of students’ social activities refers to the analysis of students’ social network to describe the relationship between students and students, students and teachers, or students and learning resources, and their respective attributes and characteristics. The analysis results can support kinds of educational applications, such as dividing the students into groups. Constructing the educational knowledge map is a method to establish the relationship between knowledge and learning resources. High quality knowledge maps in teaching and educational activities can help teachers and students more accurately understand the relationship between knowledge and better master efficient learning skills. However, as a new research direction, educational knowledge maps are developing slowly, and large-scale, high-quality educational maps are sorely lacking. Therefore, how to construct the knowledge map of general education or special education combined with a wide range of educational data is an urgent problem to be studied.

To sum up, as a novel research direction, EDM has rich research contents and diverse research methods [20]. Personalized learning is a pivotal research topic of EDM. The present work studies three important issues related to personalized learning, namely learning resources, learners, and learning strategies. Moreover, the deep learning algorithm is introduced and applied to the education of western music history to help students improve their learning efficiency.

### Research on personalized recommendation

Chiu et al. (2021) proposed in the study that the rapid development of the IoT had a profound impact on the acquisition of information. Users can select information according to their preferences and needs, but there are still some data that cannot be obtained by users. Therefore, the personalized recommendation system can eliminate this shortcoming. The personalized recommendation system can connect and filter the information in the system, and recommend appropriate information for users. The personalized recommendation system has important application value in data processing, which is very worthy of study [21]. It is essential to analyze the principle of traditional recommendation system for realizing personalized recommendation of learning resources. Based on this basic goal, the theoretical foundations can be roughly divided into the following three categories: cognitive diagnosis, the principle analysis of the traditional recommendation system, and the research on reinforcement learning based on education.

The research of cognitive diagnosis relies on online learning. The principal goal of the online learning system is to let students learn as much knowledge as possible [22, 23]. One research focus is to reasonably connect learning resources with students’ knowledge state. Therefore, it is necessary to carry out cognitive diagnosis on individual students to understand the students’ understanding level and cognitive state of a certain kind of knowledge, to effectively construct the goal of personalized recommendation. As a typical representative of the new generation of measurement theory, cognitive diagnosis can help students evaluate and analyze micro knowledge at the individual level. The measurement theories put forward by researchers in related fields contain classical measurement theory, generalization theory, and item response theory. Fig 2 reveals the knowledge example of cognitive diagnosis.

**Fig 2:** Knowledge example of cognitive diagnosis.

In traditional tests, teachers can only investigate students’ learning status through the test scores, but it is difficult to accurately figure out every detail for students with the same score level [24]. In contrast, through the knowledge example of cognitive diagnosis shown in Fig 2, even if the scores are the same, if the characteristics of the exercises of students are different, the teacher can intuitively see the student’s mastery of a certain knowledge point. Different exercise characteristics and scores can more finely reflect students’ understanding of specific knowledge details. The cognitive diagnosis can be expressed as Eq (1).


$$P(M_{\mathrm{ji}}=1|\theta_{j},a_{j},b_{j})=b_{i}^{1-\Pi_{ji}}a_{i}^{\Pi_{ji}},\Pi_{\mathrm{ji}}=\prod_{n=1}^{n}\theta_{jn}^{qin},$$ (1)

In Eq (1), *n* represents the total number of knowledge points included in the test, *a*_*j*_ and *b*_*j*_ refer to knowledge points that students are uncertain about or answer wrongly, respectively, *θ*_*j*_ signifies the knowledge vector, and *q*^*i*^ denotes the knowledge point vector that has been practiced. Moreover, Π_*ji*_ represents the knowledge mastery level of No. *j* student to knowledge point *i*.

Personalized recommendation is a feasible way to implement personalized learning in the online learning system. On the one hand, recommending appropriate learning resources can save time and improve learning efficiency for students, since it eliminates the need to search for the required content in a rich repository. On the other hand, reasonable recommendations can help improve students’ learning experience. In the traditional recommendation system, the recommendation algorithm is the core part of the project recommendation system and the focus of research. The accuracy of the recommendation result of a project recommendation system is directly related to the selection of recommendation algorithm [25, 26]. The commonly used recommendation algorithms in related research fields can be roughly divided into four types, i.e., the content-based recommendation algorithm, memory collaborative filtering recommendation algorithm, model collaborative filtering recommendation algorithm, and hybrid recommendation algorithm. The rationale behind the content-based recommendation algorithm mainly comes from information retrieval and information filtering. The so-called content-based recommendation is to recommend items that the user has not contacted according to the user’s past browsing history. The content-based recommendation method can be explained according to the heuristic method and model-based method. The heuristic method is to let users use experience to define relevant formulas, verify the calculation results of the formulas in accordance with actual results, and constantly modify the formulas to achieve the final goal. The model-based method takes historical data as the data set, and trains the model based on the data set. The keyword is used as the vector representing the user’s characteristics, and the keyword with the highest weight of the recommended element is used as the feature attribute of the recommended element. The two closest vectors (the user’s feature vector score is the highest) are recommended to the user [27, 28]. The cosine method is usually used to calculate the cosine value of the angle between user feature vector and recommended feature vector to determine the similarity between the two vectors. Fig 3 demonstrates the basic flow of content-based recommendation algorithm.

**Fig 3:** Flow of content-based recommendation algorithm.

In addition, there are the memory collaborative filtering recommendation algorithm, model collaborative filtering recommendation algorithm, and hybrid recommendation algorithm. Due to space limitations, these algorithms are not discussed in detail here. Traditional recommendation algorithms have produced many in-depth research results, but they usually model behavior activities to obtain a surface relationship between users and products, such as the linear relationship. However, in the real world, behavioral decision-making is often affected by multiple factors, and the interaction of behavior is also complex and diverse. Only linear expressions of the relationship between the two cannot meet the needs [29, 30]. Therefore, in the present work, the deep learning algorithm is applied to the education field to meet the learning needs of students.

Through reinforcement learning, the model can run in the context of the environment, and feedback can optimize the long-term behavior strategy based on income. The latest research in educational psychology combines the results of cognitive diagnosis and reinforcement algorithm learning experiments with topic recommendation personalization. However, the existing research has the following limitations. First, the existing research usually contains excessively complicated calculations and formulas. Second, the transfer function needs to be evaluated in the state action space containing all query items. Third, the memory for storing and maintaining the algorithm needs to be set. However, because the online learning system has many topic resources, it is impossible to estimate all the recommended actions. Therefore, these algorithms ignore the process factors in learning behavior and only match the current students’ learning state.

### Personalized recommendation system based on deep learning algorithm

The recommended system should have the following functions to realize the targeted recommendation of learning resources required by students. First, the recommendation system needs to recommend appropriate topics to students according to the algorithm, to avoid artificial query of students, and improve learning efficiency [31, 32]. Second, the recommendation system needs to provide an open and autonomous learning environment, which can meet the adaptive interaction between students and the system. Thirdly, the system should utilize machine learning and data mining algorithms to analyze a wealth of learning interactive data of students, to generate appropriate topic recommendations. Among them, the core technical challenge is how to design the optimal recommendation strategy to ensure that the most appropriate topics and resources can be recommended to students at the right time.

Therefore, a personalized recommendation system based on Deep Reinforcement Exercise (DRE) algorithm to realize the above functions. Fig 4 shows the basic architecture of the system.

**Fig 4:** Basic architecture of the personalized recommendation system based on DRE algorithm.

As shown in Fig 4, a targeted personalized recommendation system should have an adaptive adjustment recommendation mechanism. The recommendation system framework reported here includes three learning objectives of online topic recommendation. (1) Review and investigation: the fundamental objective of personalized topic recommendation is to obtain as much knowledge as students need. The referral process can not only enable students to find and fill vacancies in time and identify “strange” knowledge, but also acquire new knowledge at the right time, even if some knowledge is incomplete. According to Fig 4, student 1 who makes a mistake about a certain knowledge point in the second step would receive relevant knowledge recommendations in the third step. When the student can answer the question about the knowledge point correctly, the system will recommend new knowledge topics in the fourth step. (2) Smoothness of difficulty: the difficulty of recommended questions should not change drastically, because students’ knowledge learning process is gradual. For example, it is unreasonable to recommend college math problems to pupils who have just learned addition and subtraction. Therefore, the recommendation process needs to adaptively adjust the algorithm to make the difficulty of the recommended topics smoother. For example, for student 2 in Fig 4, if the recommended topics are relatively simple or familiar knowledge that he has mastered, the recommendation effect will not be satisfying. (3) Participation: the concept of participation is relatively abstract. In short, it is a vital factor to maintain students’ learning enthusiasm, and it is very important in the online learning environment. For example, the system recommends excessively difficult topics to student 3 in Fig 4, resulting in students’ lack of sense of participation and loss of interest in learning. The present work uses the off-line strategy learning algorithm to optimize recommendation strategies from off-line student data. This algorithm employs an experimental storage system to represent the two recent data experiments. The following algorithm implements two independent networks, namely the estimation network and target network. Therefore, as the difference of learning parameters decreases, the stability of the algorithm is guaranteed. These two strategies ensure the dynamics of students’ historical records. The integrated multi-functional reward function allows DRE to adjust its strategy. As an independent model algorithm, DRE can use data offline for policy learning.

In the above structure, the definition of review and survey objective can be written as Eq (2).


$$r_{1}=\{\begin{array}{l} a_{1},if,b_{t}=0,and,k_{t+1}\cap k_{t}=\emptyset \\ a_{2},i,k_{t+1|}\backslash \{k_{1}\cup k_{2}\cup \ldots \cup k_{t}\}\neq \emptyset \\ 0,else. \end{array}\}$$ (2)

In Eq (2), *a*_*1*_ represents the penalty function, *a*_*2*_ refers to the excitation function, *b*_*t*_ indicates the comprehensive learning status, and *k*_*t*_ stands for knowledge concepts.

The smoothness of difficulty is presented in Eq (3).


$$r_{2}=f(m_{t+1},m_{t})=-{\left(m_{t+1}-m_{t}\right)}^{2}$$ (3)

In Eq (3), *f*(m_*t*+1_,m_*t*_) denotes the negative square root of two numeric values. The larger the value, the closer the difficulty is. Besides, m_*t*+1_,m_*t*_ indicates the recommended topic and the topic to be recommended.

The participation is expressed as Eq (4).


$$r_{3}=1-|g-\varphi (s,N)|,\varphi (s,N)=\frac{1}{N}\sum_{i=T-N}^{T}P_{i}$$ (4)

In Eq (4), *g* represents the learning objective factor, N indicates the number of learning records, and *φ*(s,N) means students’ usual performance.

According to the above three sets of definitions, the final return coefficient can be expressed as Eq (5).


$$r=a_{1}\times r_{1}+a_{2}\times r_{2}+a_{3}\times r_{3},\;\{a_{1},a_{2},a_{3}\}\in [0,1]$$ (5)

In Eq (5), *a*_1_ represents the penalty function, *a*_2_ refers to the excitation function, *a*_3_ expresses the adjustment function, *r*_1_ accords to the coefficient of review and survey target, *r*_2_ stands for the coefficient of difficulty smoothness, and *r*_3_ stands for the coefficient of participation.

Fig 5 demonstrates the personalized recommendation method based on the DRE algorithm.

**Fig 5:** Personalized recommendation method based on the DRE algorithm.

The present work further optimizes the personalized recommendation method based on the DRE algorithm shown in Fig 5. Specifically, the Exercise Question Networks (EQNs) is introduced to estimate the state of students, and then the system recommends appropriate topics according to the estimation results. Here, two kinds of EQNs, Exercise Question Network of Markov (EQNM) and Exercise Question Recurrent Neural Network (EQNR), are employed. Figs 6 and 7 show the basic structure of these two networks.

**Fig 6:** Structures of Exercise Question Network of Markov.

**Fig 7:** Structures of Exercise Question Recurrent Neural Network.

As shown in Figs 6 and 7, students’ knowledge mastery level is perceived through EQNM and EQNR. Here, the combination of the DRE algorithm with EQNM is called DREM, and the integration of the DRE algorithm and EQNR is denoted as DRER.

### Training parameter settings and data source

The network parameters are initialized in the training process. The penalty factor is set to 0.9, the review memory size in algorithm Z = 500, and the batch size is 32. The experimental running environment is a Linux server with a CPU of 4-core 2.0GHz Intel Xeon E5-2620, and the GPU of TeslaK20m. This experiment uses two data sets, i.e., Math and History. The data set is provided by http://zx.zhixuekt.com of IFLYTEK CO., LTD, which is an online learning system developed for self-study. The system encourages students to ask questions, and then students answer them and get results. The system allows students to refer to “clues” and submit answers repeatedly. Hence, in this scenario, the data only records the students’ initial response to ensure fairness. This data set has deleted the data of students with less than 10 learning records and subjects that have never been studied from the preprocessing link, and it contains multiple knowledge archives.

## Results and discussion

### Analysis of experimental results on the rationality of learning objectives

To verify the rationality of the three learning objectives proposed above, namely review and investigation, smoothness of difficulty, and participation, the learning data of students is deeply analyzed, and the analysis results are shown in Figs 8 and 9.

**Fig 8:** Average concept coverage analysis results.

**Fig 9:** Difficulty analysis results.

According to Fig 8, the knowledge concept coverage of the long session unit is higher, indicating that students are willing to learn more knowledge. Therefore, recommendations need to consider exploring new knowledge to keep students interested in learning. Fig 9 shows the difference in the difficulty of two consecutive learning topics in each conversation unit. The line chart shows the proportion of records with difficulty difference of more than 0.4 in the conversation (it is assumed here that if the difficulty difference of two consecutive questions exceeds 0.4, the difficulty changes sharply). From Fig 9, the difficulty difference of the short session unit is large, while the long session unit has a smoother topic difficulty record. During the test, students tend to choose simpler or more difficult topics for long-term learning. In summary, the three groups of learning objectives reported here, namely review and investigation, smoothness of difficulty, and participation, have a close relationship with the learning effect of students.

### Comparison results of recommended accuracy of recommended algorithms

The offline experiment of the accuracy of the recommendation algorithms is conducted according to the learning log of students. The log data is static and contains only the student scores of the investigated subjects. Consequently, it is impossible to make sequence recommendations in the offline experiment because feedback on real-time recommendation cannot be obtained from offline data. Moreover, it is not possible to document the benefits of the various learning objectives provided above. Therefore, a single point recommendation target is adapted to evaluate the accuracy of the DRE algorithm in off-line experimental scenario. The evaluation index is the common Top@k ranking index for evaluation. The experimental results are shown in Figs 10 and 11.

**Fig 10:** Comparison of accuracy rates of recommended algorithms in math dataset offline experiments (IRT refers to the Item Response Theory algorithm, PMF represents the Probabilistic Matrix Factorization algorithm, FM represents the Factorization Machine algorithm, DKT represents the Deep Knowledge Tracing algorithm, DKVMN represents the Dynamic Key-Value Memory Network, DQN represents the Deep Q Network).

**Fig 11:** Comparison of accuracy rates of recommended algorithms in History dataset offline experiments (IRT refers to the Item Response Theory algorithm, PMF represents the Probabilistic Matrix Factorization algorithm, FM represents the Factorization Machine algorithm, DKT represents the Deep Knowledge Tracing algorithm, DKVMN represents the Dynamic Key-Value Memory Network, DQN represents the Deep Q Network).

As shown in Figs 10 and 11, the two data sets are operated in DRER and DREM. The results show that DRE can interactively learn the best strategies of students’ behavior and put forward specific suggestions. Besides, the combination of complex EQNs (EQNR and EQNM) makes DRER and DREM algorithm possible, which are better than the simple DQN algorithm. This phenomenon proves that the theme evaluation proposed here is effective. Capturing rich information in the dynamic learning process of students can improve students’ health level and accurately represent it. Moreover, DRER is better than DREM, indicating that the network is built based on cyclic sequence. Since EQNR can track the long-term dependence characteristics of students’ learning history, it improves the performance of recommendation. In addition, it can be confirmed that the effect of DRER on Math data set is not as good as that on History data sets. Although DREM has a simple structure and lacks data, it is still superior. In terms of the average record length of the data set, the average record length of the Math data set is 24.5, which is much smaller than that of the History data set. Finally, the performance of conventional methods (IRT, PMF, and FM) is lower than that of deep learning algorithms (DKT, DKVMN) and reinforcement learning algorithms (DQN, DREM, and DRER). The reason for this phenomenon is that the existing algorithms cannot accurately model the learning process that ignores the dynamic characteristics of students’ learning behavior, which affects the recommendation results. In short, the DRE model perfectly simulates students’ research performance and information about related files, to produce accurate recommendation results.

The operation process of three learning objectives (i.e., the reasonable return function of review and investigation, smoothness of difficulty, and participation) is verified by the recommended results of observation experiments. The operation process curve of review and investigation is shown in Figs 12 and 13.

**Fig 12:** Review job flow curves.

**Fig 13:** Investigate job flow curves.

Figs 12 and 13 reveal that various stimulus coefficients are set in the DRER algorithm in the experiment. Through the observation on the cumulative coverage rate of knowledge concepts in the recommendation process, it shows that in the Math data experiment, the values of each detection parameter are lower than those in the History data experiment, and the maximum difference is about 20. Besides, there are two similar change curves of the two data detection methods. The results show that, firstly, with the progress of the recommendation, the cumulative range of recommended topics of DRER algorithm increases. The higher the DRER incentive factor, the wider the range of knowledge recommended by the numerical algorithm. Therefore, combined with the learning objective of the review and investigation provided here, the DRE framework can explore different knowledge concepts in the recommendation process. In addition, the higher the value of the incentive factor, the more important the exploration factor.

Firstly, the DRE algorithm is used to set various learning objectives. g = {0.2, 0.5, 0.8} simulates the needs of three students. According to the DRER framework, it is recorded in the experiment. Figs 14 and 15 reveal the comparison results of the income of smoothness of difficulty and participation.

**Fig 14:** Difficulty benefit comparison.

**Fig 15:** Participation benefit comparison.

Figs 14 and 15 indicate that, from the comparison results of difficulty smoothness and participation income suggested here, the difficulty value of DRER algorithm changes greatly in Math data experiment. The highest is about 0.98, the lowest is about 0.24, and the span of difficulty change under three coefficients is more than 0.4. In the “History” data experiment, the difficulty change span is 0.2 for the DRER algorithm under the three coefficients. The DRE recommendation algorithm has two advantages. First, it can adaptively control the difficulty target of recommended questions. In this process, the difficulty of recommendation problems can be adjusted adaptively. Secondly, the learning objective of participation allows students to set different learning goals and choose questions with different difficulty ranges. The results show that in most courses recommended by DRER, the difficulty level of questions is relatively stable, so the fluency goal can effectively control the difficulty and reliability of the recommendation process. However, in the experiment of the Math data set, the recommendation result of step 10 is not good, and the difficulty level varies greatly. The reason for this phenomenon is that the DRER algorithm still cannot accurately simulate students’ knowledge state at the beginning of recommendation, which affects the stability of recommendation results. In addition, if the goal is set relatively high, the problems that students can challenge are difficult, and the DRER algorithm will select more difficult topics for recommendation accordingly. From the results, most students answer the recommended questions incorrectly, indicating that the results of the participation experiment of the recommendation algorithm meet the expectations. Based on the above two results, the DRE recommendation algorithm can adapt to different learning needs and customize the recommendation results.

### Discussion on the results

The research results suggest that the existing algorithms are relatively lacking in all aspects, and the DRER algorithm proposed here has advantages in all aspects. Initially, in the aspect of learning modeling, ignoring the dynamic characteristics of students’ learning behavior, the average record length of DRER algorithm is much higher than that of the existing algorithm, with an average of 24.5. Then, through the observation of the cumulative coverage of knowledge concepts, the values of Math and History data experiments differ by about 20, but the change curves of the two are very similar, which increase with the increase of the incentive factor. The DRE recommendation algorithm can improve the coverage of knowledge accumulation. Finally, in terms of difficulty recommendation of test questions, the difference between the two data experiments is large. The DRE recommendation algorithm can adapt to recommend various difficult test questions according to the characteristics of students, and is more adaptable than the existing algorithm. It proves that the algorithm proposed here in the teaching research of western music history through DL algorithm can adapt to various teaching conditions and provide more comprehensive teaching effect for students.

## Conclusions

The teaching mode under the environment of Internet of Things has changed greatly, but improving the teaching level and perfecting the teaching mode is still the primary task in the education field, and the teaching of western music history is also facing the same situation. Therefore, at first, the present work summarizes the current situation of the changes in teaching reform under the background of the IoT, analyzes the related work of personalized recommendation research, and then introduces the DL algorithm, which is applied to the learning of western music history to help students improve learning efficiency. What is proposed is a personalized recommendation method based on DRE algorithm. The recommendation accuracy and performance of the recommendation algorithm are verified by offline and online experiments. The purpose is to improve the teaching mode of western music history in the IoT environment. The results show that the proposed personalized learning resource recommendation method based on DRE still has good stability under various training data scales. The difficulty of recommended questions can be adjusted adaptively according to the characteristics of students to meet the individualized needs of western music history education. It can provide accurate teaching guidance for students, recommend moderate difficulty training questions for students according to their own characteristics, strengthen students ’ autonomous learning ability, and improve teaching level. The present work study can improve students’ learning effect to a greater extent and improve the teaching mode of western music history. Although some achievements have been made, there are still some limitations. Firstly, due to the limited research funding and research level, the research design field is not wide, which brings certain errors to the results. Secondly, the research on DL algorithm still stays at the shallow level. In future research, the above two points will be improved to make the results more accurate and improve the persuasiveness of the article.

## Supporting information

S1 Data (XLSX)

## References

[1] BarlowH, HerbertT. Introduction Listeners in Music History: Studying the Evidence. Nineteenth-Century Music Review, 2020; 17(3):343–357.

[2] Hilpert JC, Marchand GC. Complex systems research in educational psychology: Aligning theory and method. Educational Psychologist, 2018; 53(3): 185–202. doi: 10.1080/00461520.2018.1469411 31431794PMC6701846

[3] HaryatiS. The Effectiveness of the Process Oriented Guided Inquiry Learning (POGIL) Model in Educational Psychology Learning. International Journal of Pedagogy and Teacher Education, 2018; 2(2): 375–388.

[4] HuangX. Aims for cultivating students’ key competencies based on artificial intelligence education in China. Education and Information Technologies, 2021; 26,5 127–5147.

[5] LeeM. An analysis of the effects of artificial intelligence on electric vehicle technology innovation using patent data. World Patent Information, 2020; 63(2019):102002.

[6] Edwards BI, Cheok AD. Why not robot teachers: artificial intelligence for addressing teacher shortage. Applied Artificial Intelligence, 2018; 32(4): 345–360.

[7] DanielJ. Sección Femenina: Documenting and Performing Spanish Musical Folklore During the Early Franco Regime (1939–1953). Music and Letters, 2019; 24(3):3.

[8] Shin SA Study on the Framework Design of Artificial Intelligence Thinking for Artificial Intelligence Education. International Journal of Information and Education Technology, 2021; 11.9:392–397.

[9] Torshizi MD, BahramanM. I explain, therefore I learn: Improving students’ assessment literacy and deep learning by teaching. Studies In Educational Evaluation, 2019, 61:66–73.

[10] GuX, O’ConnorJ, NgJ. Worlding and new music cultures in Shanghai. City Culture and Society, 2019; 19:100286.

[11] ThomasH. The effect of education on poverty: A European perspective. Economics of Education Review, 2021; 83:102124.

[12] WhiteP B. Using Data Mining for Citation Analysis. College & Research Libraries, 2019, 80(1):76–93.

[13] Ham MeL S. Music, the Realist Conception of Art and the Materialist Conception of History. twentieth century music, 2019; 16(1):33–50.

[14] CrystalG, SotiriaP. EFL Teacher Education in Finland: Manifestations of Professional Agency in Teacher Educators’ Work. Scandinavian Journal of Educational Research, 2021; 65(4):552–568.

[15] Mavezera TF, GwirayiC, KufakunesuM. Attitudes of Primary School In-Service Undergraduate Student Teachers towards Educational Psychology in Zimbabwe. International Journal of Arts Humanities and Social Sciences Studies, 2019; 4 (8): 9, 14.

[16] CastillaD, BotellaC, MirallesI, et al. Teaching digital literacy skills to the elderly using a social network with linear navigation: A case study in a rural area. International Journal of Human-Computer Studies, 2018; 118: 24–37.

[17] WangT, ZhiF, YutongL U, ZhangJ. Effect of Dong Chorus on the executive function of Dong high school students. Acta Psychologica Sinica, 2019; 51(9):1040.

[18] MoscatoD. The metanarrative of rural environmentalism: Rhetorical activism in Bold Nebraska’s Harvest the Hope. Public Relations Inquiry, 2019; 8(1):23–47.

[19] MusicKennerley D., Politics, and History: An Introduction. Journal of British Studies, 2021; 60(2):362–374.

[20] RastgouM, BayatH, MansoorizadehM, Gregory AS. Estimating the soil water retention curve: comparison of multiple nonlinear regression approach and random forest data mining technique. Computers and Electronics in Agriculture, 2020; 174: 105502.

[21] ChiuM C, HuangJ H, GuptaS, et al. Developing a personalized recommendation system in a smart product service system based on unsupervised learning model. Computers in Industry, 2021, 128(10):103421.

[22] GrishchenkoA V, KruchekV A, KurilkinD N, KhamidovO R. Diagnostics of the technical condition of rolling bearings of asynchronous traction motors of locomotives based on data mining. Russian Electrical Engineering, 2020; 91(10): 593–596.

[23] LinM, ChenX, WangZ, WangD, Zhang JL. Global profiling and identification of bile acids by multi-dimensional data mining to reveal a way of eliminating abnormal bile acids. Analytica Chimica Acta, 2020; 1132:74–82. doi: 10.1016/j.aca.2020.07.067 32980113

[24] ChangM, D’AnielloG, GaetaM, OrciuoliF, SimonelliC. Building Ontology-Driven Tutoring Models for Intelligent Tutoring Systems Using Data Mining. IEEE Access, 2020; 8(1):48151–48162.

[25] HsrpdA, FukudaP T, TamakiP Y, HanashiroB K, KspdC, EurpdD. Computerized data mining analysis of keywords as indicators of the concepts in aha-bls guideline updates. The American Journal of Emergency Medicine,2020; 38(7), 1436–1440. doi: 10.1016/j.ajem.2019.11.045 31866248

[26] LiG, DuanZ, LiangL, ZhuH, HuW. Outlier data mining method considering the output distribution characteristics for photovoltaic arrays and its application. Energy Reports, 2020; 6:2345–2357.

[27] LiangW. Scene art design based on human-computer interaction and multimedia information system: an interactive perspective. Multimedia Tools and Applications, 2019; 78(4): 4767–4785.

[28] ChenM. The impact of expatriates’ cross-cultural adjustment on work stress and job involvement in the high-tech industry. Frontiers in psychology, 2019; 10: 2228. doi: 10.3389/fpsyg.2019.02228 31649581PMC6794360

[29] LiT, WangZ, LiuJ. Evaluation method for impact of jamming on radar based on expert knowledge and data mining. IET Radar, Sonar & Navigation, 2020; 14(9):1441–1450.

[30] WuY, SongD. Gratifications for social media use in entrepreneurship courses: learners’ perspective. Frontiers in Psychology, 2019; 10: 1270. doi: 10.3389/fpsyg.2019.01270 31214081PMC6555126

[31] LiS, BhattaraiR, Cooke RA, VermaS, ChristiansonL. Relative performance of different data mining techniques for nitrate concentration and load estimation in different type of watersheds. Environmental Pollution, 2020; 263:114618. doi: 10.1016/j.envpol.2020.114618 33618470

[32] CalderónF, Miller EJ. Bridging the knowledge gap in ride hailing service provision with human-driven fleets: A data mining approach. Procedia Computer Science, 2020; 170: 673–680.

